# Design of a Smart Elbow Brace as a Home-Based Rehabilitation Device

**DOI:** 10.1155/2022/3754931

**Published:** 2022-06-16

**Authors:** Ramadhan Rashid Said, Wang Quan Yong, Md Belal Bin Heyat, Liaqat Ali, Song Qiang, Arif Ali, Hafiz Tayyab Rauf, Zhe Wu

**Affiliations:** ^1^School of Life Science and Technology, University of Electronic Science and Technology of China, Chengdu, China; ^2^IoT Research Center, College of Computer Science and Software Engineering, Shenzhen University, Shenzhen, China; ^3^International Institute of Information Technology, Hyderabad, Telangana 500032, India; ^4^Department of Science and Engineering, Novel Global Community Educational Foundation, Hebersham, NSW 2770, Australia; ^5^Department of Electrical Engineering, University of Science and Technology Bannu, Bannu, Pakistan; ^6^Chengdu Technology University, Chengdu, China; ^7^Department of Computer Science, University of Science and Technology Bannu, Bannu, Pakistan; ^8^Centre for Smart Systems, AI and Cybersecurity, Staffordshire University, Stoke-on-Trent, UK

## Abstract

Poststroke and traumatic elbow injuries are the most common cause of elbow stiffness, which results in loss of functional range of motion (ROM). Various studies support early mobilization of the elbow joint after injury or after surgery to reduce risks of elbow stiffness development. After hospitalization, patients are required to follow a long-term rehabilitation program during home recovery. Still, most patients do not adhere to their clinical therapy schedule due to either rehabilitation cost, social obligations, negligence, or lack of inspiration. Moreover, the numbers of therapists and assessment equipment are insufficient. This study introduces a smart elbow brace (SEB) as a home-based rehabilitation device that reduces regular in-patient rehabilitation costs and therapist workload and motivates patients to comply with the rehabilitation program that enhances the achievement of rehabilitation goals. Our device has two active degrees of freedom (2-DoF) that allow extension, flexion, pronation, and supination elbow motions. An extra sliding joint between forearm and wrist is added, which helps dump forces concentration at the elbow joint during extension-flexion movement. Mechanical design requirements, motion-tracking systems, and serious game development are described. The feasibility of a proposed SEB device is tested with five healthy subjects playing developed serious games with the device. The results show that subjects can attain maximum and minimum angles of flexion-extension and pronation-supination motion designed for elbow stiffness rehabilitation. The SEB device will be beneficial and be used at home as a complementary tool to support elbow stiffness rehabilitation during long-term home recovery.

## 1. Introduction

Elbow joint is crucial in human activities of daily living (ADL); such activities are like being able to touch every part of the body, reaching an object in space, holding staffs, and offering exactness in both closed and open kinetic chain work. A stable, pain-free joint with sufficient strength and range of motion is required for proper elbow function [1]. Poststroke and elbow injuries are the most common cause of elbow stiffness development, which results in loss of functional range of motion (ROM). Studies [2, 3] reported that prolonged immobilization of an elbow joint following poststroke or elbow injuries results in elbow stiffness and can cause extensive impairment of upper limb function. Loss of extension-flexion or pronation-supination ROM embodies a severe limitation on ADL, which makes an individual's life difficult [4, 5]. Sojbjerg [1] has defined elbow stiffness as a flexion less than 120 degrees or extension greater than 30 degrees of full ROM of an elbow joint. It also can be a loss of range of motion pronation-supination of lower than 100 degrees. Studies [6, 7] defined that functional ROM of a typical elbow joint permits an extension of 0 degrees with flexion of about 145 degrees and pronation and supination motion of 80 degrees and 75 degrees, respectively, but individual variability should be considered. The study by Morrey et al. [8] described that functional ROM is required for an individual to conduct 90% of routine daily activities. Elbow flexion-extension should be at least 100 degrees, ranging from 30 degrees to 130 degrees, with forearm pronation-supination of 100 degrees, ranging from 50 degrees of pronation to 50 degrees of supination, but this does not relate to sports and work range of motion.

Currently, with the use of splints (mechanical braces), clinical rehabilitation has shown promising results in reducing the risk of elbow stiffness development risks, hence restoring functional ROM of the elbow joint [9]. Splints use forces imposed on the muscles to load tissues to a boom range of the muscles' plasticity when there is no heterotopic ossification. Two types of available splints are commonly used. Dynamic splints [9, 10] employ stress reduction principles to escalate the range of motion in the tissues. Reducing stress on the muscles is the more rapid and dependably causative factor of plastic distortion. Dynamic splints normally use elastic rubber or springs that need to be changed often as they elongate. Again, these splints are timely used for substantial hours in the day. Static progressive braces are preferred because they tolerate biological alteration of the tissue by employing stimulation interchanged with a break [11]. In the ultimate degrees of flexion, compression forces are employed on the humeroulnar joint, while distraction forces are employed in the ultimate degrees of extension.

Problems emerge after hospitalization, following poststroke or elbow injuries that require a minimum protection period in which the joint should be immobilized in a cast. Then, it is crucial to lengthening ROM for the joint to avoid elbow stiffness development. Since stiff elbow takes a long time to improve, from 6 months to 12 months [9], the patient should proceed with exercise after hospital discharge, requiring to follow a long-term rehabilitation program during home recovery. Due to the various challenges facing these mechanical devices, alternative ideas for stiff elbow training programs that involve smart wearable device technology for recording patients' movements have been developed in recent years [12–15]. However, these wearable devices require supervision; they are expensive, offer no motivation, and cannot be used outside the clinical environment. The majority of patients fail to follow their clinical therapy schedule due to either rehabilitation cost, social obligations, negligence, or lack of inspiration [13, 16, 17]. Moreover, other studies [18–20] reported an insufficient number of therapists and assessment equipment. Being unable to attend clinical rehabilitation schedule as per therapists' instructions during home recovery after being discharged from hospital leads to other complications at the elbow joint, especially loss of ROM due to elbow stiffness development; in the end, very few patients regain functional ROM. Several authors [18–22] reported that home-based rehabilitation shows a higher satisfaction rate and better results.

Maintaining patients' motivation is one of the key elements for patients to attend all prescribed rehabilitation programs by the therapist during home recovery. Serious game applications for healthcare have become more prevalent, and there are now a large number of them available [23]. Some of the popular commercial gaming systems have shown rehabilitation potential in upper limb rehabilitation; such games are the Nintendo® Wii remote, Microsoft® Kinect, and Sony® PlayStation Eye toy [24–30]. Indeed, serious games help create a motivating environment for rehabilitation that provides physical meaning in rehabilitation exercises. However, commercial video games are difficult for the patient to engage with because they were designed for normal healthy users; also, these games are costly and are vulnerable to ambient light [31] and camera vision [14, 32].

Thus, a home-based rehabilitation with serious games designed for a specific patient's condition is a promising option as a complementary tool to support elbow stiffness rehabilitation during long-term home recovery. However, despite the effort made for home-based rehabilitation training aids projects, there is still no reliable design for poststroke patients who suffer from stiff elbow. Hence, developing a smart elbow brace as a home-based elbow joint training aid for elbow stiffness patients is necessary to enhance their recovery.

In this study, we introduce the novel smart elbow brace (SEB) (see Figure 1) designed for poststroke or any other elbow complications from elbow injuries that require early rehabilitation to prevent elbow stiffness development, ensuring comfort and safety and rehabilitation adherence to the patient. SEB provides four innovative design solutions:

1. A lightweight and compact home-based rehabilitation device that motivates and assesses changes beyond the clinical environment.
2. A two-degree-of-freedom (2-DoF) elbow brace model that matches the kinematic structure of an elbow joint and unloads the elbow articulation from undesired loads.
3. A reliable device that provides smooth motion pain-free by ensuring the exact alignment of the human arm and SEB joint axes.
4. Development of serious games that are specifically for elbow stiffness rehabilitation.

## 2. Design Methods

The detailed design of SEB developed in this paper is presented in Figure 2. It consists of the elbow brace that allows both extension-flexion and pronation-supination ROM, the IMUs MPU6050 motion sensor that tracks the movement of the elbow joint and sends signals to the computer through the Bluetooth module, and the serious games (computer games) as the motivational tool that decode signals received into playable games for adherence of rehabilitation program as well as promoting rehab individualization.

The system architecture of the developed SEB is presented in Figure 3. During rehabilitation, the type of game, movement, time, and speed must be configured according to the therapist's instructions. The motion sensor then records the movement of an elbow joint and transmits the tracking signals to the playable game through a Bluetooth module. The game's scores will be recorded on a user's personal computer at the end of the game, where all data can be emailed to the therapist for monitoring and progress evaluation.

The intended primary functions of the designed elbow brace are to protect an elbow joint at any stage, avoid elbow stiffness development by providing joint mobility during early rehabilitation, and imitate a standard rehabilitation training program. Four independent factors were well thought out as the main requirements for the design of an elbow brace to meet these functions, which are as follows:

1. To accommodate a wide range of patients with different upper limb size.
2. To support the upper limb during rehabilitation.
3. Mobilization of a wide range of elbow kinematic.
4. To ensure comfort and safety during rehabilitation.

### 2.1. Mechanical Elbow Brace Design

The development of the mechanical elbow brace was designed using SolidWorks version 2019 software so as the finite element analysis (FEM) of the developed brace. The general hardware design requirements of the brace are according to the anatomical and kinematic structure of the elbow joint.

#### 2.1.1. Standardization

We considered the differences in anthropometric parameters of people's bodies in our design. The elbow brace was designed in such a way that it should be able to cover 95% of the population (adults), based on [17, 33, 34] anthropometric data presented in Table 1. To ensure that the forces acting on the forearm are well supported naturally and efficiently, the forearm splint should be positioned on the lower arm's and hand's center of mass (31.8%). The lower forearm frame length is calculated as follows:

(1) $$\begin{array}{c} l_{\mathrm{FS}}=\;l_{\mathrm{FL}}\mathrm{xCOM}\text{,} \end{array}$$

where *l*_FS_ is the position of the forearm splint (m), *l*_FL_ is the length of the hand (m), and COM is the lower arm and hand center of mass (%).

The calculated position of the forearm splint will vary between 0.14 m and 0.17 m based on the human anthropometric data in Table 1, providing a higher momentum to minimize the supporting force operating on it. Because the upper arm splint was effective enough to be placed in the middle of the upper arm frame, its position will range from 0.17 to 0.2 m. The biceps width will vary from 9 to 13 cm, and the breadth of the forearm will range from 7 to 11 cm, while the width of the forearm wrist will range from 7.4 to 8.2 cm, according to Table 1.

#### 2.1.2. Total Load Supported

During rehabilitation, especially at the strength training stage, a patient would be required to carry a certain amount of weight, such as a ball of 1 kg. Therefore, knowing the total load that the brace can support is essential to avoid any mechanical failure. The elbow brace must sustain the forearm's weight plus the weight carried by the forearm plus its weight to prevent any failure, as shown in Figure 4. Therefore, the total load was calculated as follows:

(2) $$\begin{array}{c} F=\mathrm{MXg}, \end{array}$$

(3) $$\begin{array}{c} M=m_{\text{device}}+m_{\text{load}}+\;m_{\text{hand}}, \end{array}$$

where *F* is the total load, the total mass which the forearm splint has to be able to sustain is *M*, which consists of device mass (0.7 kg obtained from designed material) + hand lower arm mass (from Table 1) + carried load), and *g* is the gravitational force of the Earth equal to 9.81 m/s^2^.

Applying these figures as well as the 95th percentile anthropometric data provided in Table 1 in the total load equation above, the calculated total load was 29 N and 33 N for females and males, respectively. From the literature review [35], the total load required by the biceps during performing activities of daily living was found to exceed this range. Therefore, the above-obtained values fit the minimum requirement of the total load that the patient can exercise and wear the device daily without any disturbance or feeling tired.

#### 2.1.3. Mobilization

Structurally and functionally, the humerus and ulna of an elbow joint are considered hinge joints that allow flexion-extension motion, while the proximal radioulnar joint and humeroradial joint act as pivot joints that contribute to the movements of pronation-supination [36]. The designed elbow brace was modeled as two degrees of freedom (2-DoF) to mimic an elbow joint kinematics structure for better mobility. The total safe range of flexion-extension motion was 135 degrees, while pronation-supination motion was 100 degrees, as shown in Table 2. From various studies of the elbow joint, the length of the forearm changes during flexion-extension motion due to the shifting of an elbow joint center [37–39]. When the length of an elbow brace is rigid, it restricts the variation of the forearm length. Because of the concentration of forces at the elbow joint and friction, the user may be unable to tolerate such pain and, as a result, quit the use of the brace. A free sliding joint was added in the middle of the wrist and forearm to allow forearm length change during flexion-extension movement to relieve pain at the elbow joint. This sliding joint unloads the forces concentrated at the joint to allow smooth movement during flexion-extension motion (Figures 2 and 3).

#### 2.1.4. Safety and Comfortability

Since the brace will protect and rehabilitate the elbow joint after joint trauma or after surgery, safety and comfortability are vital features in enhancing home-based rehabilitation. The angle stopping mechanisms were incorporated to hold the elbow joint at any prescribed safe position that allows slow healing of soft tissue (Figure 5). The device was covered with a high thick pad to prevent direct skin contact with the device. Additionally, the SEB was manufactured using nontoxic lightweight nylon resins, which provide a smooth surface to avoid friction and portability. Most of its part was made to be detachable to allow easy replacement if any damage occurs.

### 2.2. Motion-Tracking System Development

The architecture of this system was made with IMUs MPU-6050 combined with a Digital Motion Processor (DMP), a 3-axis accelerometer, and a 3-axis gyroscope in the circuit board of (4 × 4 × 0.9) mm suite 6-axis. The IMU MPU6050, which has excellent accuracy, is small in size, has low power consumption, test-retest reliability, and programmability, and tolerates high shock. The class two Bluetooth module HC-05 v2.0 + EDR with 3.3 voltage uses a serial UART interface (pins RX, TX) for communications and allows the AT command. The 3.7V1800 mAh lithium polymer battery is light-weight and pliable, and provides high conductivity.

The supply voltage of 3.7 V was connected to the pin VCC of the Bluetooth module, and the VCC from the Bluetooth module was connected to the VCC of the MPU6050. The serial interface UART pins TX and RX that are connected to the RX and TX of the IMU MPU6050, respectively, are in the circuit board. The Bluetooth module is detected via the computer as HC-05 to pair the device, and then the password 1234 is entered. The computer displays a virtual COM port terminal to transmit data (COM 3 or COM 4 in our computer) from the IMU MPU6050 sensor to the game console (Figure 6).

#### 2.2.1. Motion Sensing Algorithm

*(1) Orientation Axes of Elbow Joint*. To find rotation axes of the elbow joint, the IMU MPU6050 is placed at the wrist of the forearm splint with coordinate (*x*, *y*, *z*) (Figure 7). Both rotation axes of flexion-extension (*R*_FE_) and pronation-supination (*R*_PS_) were calculated about the upper arm frame. XE stands for north, YE stands for the east, and ZE stands for the south in the Earth coordinate frame. The elbow joint coordinate frame for the forearm was described as follows: XJ, left; YJ, up; and ZJ, front, while the arm is in repose position [40].

Finding the orientation axis of the joint  *R*_FE_ about the upper arm frame, the angle of the forearm IMU about the frame of the upper arm at the first point and the last point is calculated as in [40–42]

(4) $$\begin{array}{c} R_{\mathrm{UJ}}^{f}={\left(R_{\mathrm{EU}}^{l}\right)}^{T}R_{\mathrm{EJ}}^{f}, \end{array}$$

where *f* and *l* represent the first and last points, whereas the letter *E* represents the Earth IMUs frame and *J* represents the forearm IMUs frame. The orientation matrix RXY denotes the rotation of frame *Y* in frame *X*. In the forearm IMUs frame, the orientation matrix of the last point with respect to the first point is

(5) $$\begin{array}{c} R_{\mathrm{EJ}}^{\mathrm{fl}}=\left(R_{\mathrm{EJ}}^{f}\right)R_{\mathrm{EJ}}^{l}. \end{array}$$

The ant-symmetric matrix *S*_*J*_^*fl*^ that characterizes the axis of rotation of *R*_*J*_^*fl*^ is

(6) $$\begin{array}{c} S_{J}^{\mathrm{fl}}=R_{J}^{\mathrm{fl}}-{\left(R_{J}^{\mathrm{fl}}\right)}^{T}. \end{array}$$

The orientation axis in the forearm IMUs frame is obtained from the following equation:

(7) $$\begin{array}{c} W_{J}={\left[S_{1},S_{2},S_{3}\right]}^{T}÷\sqrt{\left(S_{1}^{2}+S_{2}^{2}+S_{3}^{2}\right)}, \end{array}$$

where S1, S2, and S3 are the independent components of *S*_*J*_^*lf*^.

The same method was used to calculate the rotation axis of the elbow joint RPS to the reference of the upper arm frame. From the explanations of Instantaneous Helical Axes (IHA) [89], a least-squared method was used to obtain the optimal axes during elbow motion:

(8) $$\begin{array}{c} J\left(W_{\text{opt}}\right)=\sum_{i=1}^{10}W_{\text{opt}}-W_{i}. \end{array}$$

*(2) Calculations of Elbow Joint Angles*. The orientation IMUs data obtained during pronation-supination and flexion-extension training motion to the reference of the upper arm were used to estimate the elbow joint angle. The first point or reference position was considered when the forearm is at a 90-degree position, and the palm is at the neutral position, while the thumb points up; it is a nonsupination-pronation point.

The orientation matrix of the forearm rotation axes is given in (1) and (2). At time step *n* with relative to the Earth frame, the forearm orientation can be calculated as

(9) $$\begin{array}{c} R_{\mathrm{EF}}^{n}=R_{\mathrm{EJ}}^{n}R_{\mathrm{JF}}^{0}. \end{array}$$

The rotation axis can be represented with a skew matrix as

(10) $$\begin{array}{c} \tilde{S}=R-R^{T}=\left[\begin{array}{ccc} 0 & -S_{z} & S_{y}\\ S_{z} & 0 & S_{x}\\ -S_{y} & S_{x} & 0 \end{array}\right]. \end{array}$$

Also, it can be represented as *R*=*e*^*sλ*^, where *λ* is an angle of orientation or as

(11) $$\begin{array}{c} R=e^{\tilde{S}\lambda }=\left(1+\text{sin}\left(\lambda \frac{\tilde{S}}{S}\right)\right)+\left(1-\text{cos}\left(\lambda \frac{\tilde{S}}{S^{2}}\right)\right). \end{array}$$

Since the elbow joint has two degrees of freedom, the movement elbow joint is obtained from two repeated orientations: around *R*_FE_ axis and around *R*_PS_ axis:

(12) $$\begin{array}{c} R_{\text{joint}}=e^{{\tilde{S}}_{\mathrm{FE}}\lambda_{\mathrm{FE}}}e^{{\tilde{S}}_{\mathrm{PS}}\lambda_{\mathrm{PS}}}, \end{array}$$

where *S*_FE_ and *S*_PS_ are the antisymmetric matrices that relate to RFE and RPS, respectively, while *λ*_FE_ and *λ*_PS_ are the corresponding orientation angles.

### 2.3. Serious Game Development

The serious games (computer games) were developed using unity3D as a game engine development, and the programming language used was C#. Four rehabilitation games were designed to provide training and feedback evaluation to enhance elbow joint exercise. Each game provides a pronation-supination movement and flexion-extension movement depending on the user's preference. The game was designed so that the physical therapy done in the rehabilitation center under therapists' supervision was converted into usefully playable games. With the help of a smart elbow brace, rehabilitation training can be done at home without therapist supervision. Different levels of serious games were made to test the improvement.

Furthermore, we developed an avatar of a player (Figure 8). Before starting the game, an avatar is set such that it shows the position of the elbow. From the game setup manual (Figure 3), the avatar will show whether the type of exercise set up for exercising is correct; for example, when the patient wants to exercise flexion-extension motion with a left elbow joint, the avatar will show whether it is a correct type of motion with a right elbow joint or is wrong. At the end of the game, the scores, time used, and maximum and minimum results of angles of the joint reached are saved automatically at the user's personal computer, where all data will be sent to the therapist for progress evaluation.

### 2.4. SEB Testing

We conducted finite element analysis (FEA) on the forearm frame. The forearm was subjected to the total load acting on as calculated, and a safety factor (FoS) was added. These simulations were conducted to observe if the designed elbow brace and materials selected could withstand the stresses due to the subjected force. A total of 60N of force acted on the forearm frame distributed uniformly, and the material tested was AISI 316 annealed stainless-steel alloy (https://matmatch.com/learn/material/aisi-316-stainless-steel).

We also tested the ability of the device to provide mobilization at any stage of rehabilitation treatment. The flexion-extension and pronation-supination movements were performed, while the smart elbow brace was put on the arm. Five healthy individuals, two of them female and their mean age was 26 years old, volunteered to participate in the testing to validate the usability of our device. Participants were required to wear our smart elbow brace (SEB) on their left hand (Figure 9). Participants played the developed ball-catching game for 30 seconds with a speed of 8 m/seconds to test flexion-extension and pronation-supination ROM. All the maximum and minimum angles used to design an elbow brace, as shown in Table 2, were tested.

## 3. Results

The fundamental goal of this work is to develop a functional home-based rehabilitation tool that meets the mechanical requirements and has the potential to deliver mobilization at every stage of rehabilitation treatment during home recovery.

The results were obtained from the forearm frame. The maximum stress under a load of 60 N archived was 9.21e + 007 N/m^2^, which is far less than the yield strength of the material (Figure 10). The results indicate that the materials selected can support the total weight with the factor of safety. A factor of safety is simply defined as the ratio of the strength of a material to the expected working stress and is calculated as

(13) $$\begin{array}{c} \text{Factor of safety}=\text{ultimate strength}÷\text{actual stress.} \end{array}$$

The motion sensor signal was extracted when the participants played the game and presented in Figure 11. Participants were able to reach maximum and minimum angles designed for rehabilitation. The IMU sensor was able to detect the angles of the subject's elbow joint at an initial position (depending on starting position of the game) and reach the maximum and minimum of both flexion-extension (Figure 11(a)) and pronation-supination angles (Figure 11(b)). The MEMS MPU6050 was very sensitive to detecting the small movements of the subject's elbow joint. The digital motion processing unit onboard MEMS IMUs MPU6050 sensor corrects the shaking of an elbow joint during movement and the accumulated integration error over time.

## 4. Discussion

The paper presented shows the feasibility of implementing home-based rehabilitation for stiff elbow patients based on combining a mechanical brace, motion sensor, and computer games. SEB provides motivation and adherence to the rehabilitation training program as per the therapist's instructions.

Before creating a prototype, the general criteria of the brace design are based on the anatomical and kinematic structure of the elbow joint. According to elbow joint anatomical and kinematic studies, the elbow joint possesses two degrees of freedom (2-DoF) that allow extension-flexion motion and pronation-supination motion. The modest increase in forearm length during flexion-extension motion caused by altering the center of rotation at the elbow joint was factored into the design to minimize any misalignment between the device and the arm, which could lead to further difficulties. Regrettably, available prototypes ignore these design requirements.

The IMU MPU6050 sensor was used in this paper as a motion sensor and game controller due to its great advantages over the other motion sensors; such advantages are considered as a high accuracy motion sensor, small in size, and low power consumption that tolerates high shock, repeatability, and programmability. Furthermore, the MEM-IMUs are the most commonly used in movement tracking sensors, also are mostly wearable directly or attached to the wearable rehabilitation device to track the exercise of functional range of motion, and provide the performance of motion during upper limb rehabilitation.

Maintaining motivation is one of the main goals of home-based rehabilitation for stiff elbow patients to adhere to all prescribed training programs. The developed games were designed with different game levels to enhance patient engagement and promote the progression of elbow joint training. The designed levels are based on the speed and time setup. This means that the game's speed and time setup determines the game's level. At the beginning of the training, the therapist decides which speed and how long the patient should play a serious game. Speed and time during playing provide hierarchical order of difficulty regarding how long and fast the elbow joint can be moved to complete the task. Setup game speed starts from 1 second to 10 seconds, and playing game time starts from 10 seconds to 100 seconds.

Moreover, the results were saved on the user's personal computer at each end of the game. The saved results obtained from the game include training time, scores, speed used, and maximum and minimum angles reached for either flexion-extension movements or pronation-supination movements. The therapist can access these data for the progress evaluations and then send back information to the patient for further instructions. This method will encourage patients to stick to the prescribed training program. The development of minigames for upper limb rehabilitation using the advanced mechatronics MEMS IMUs sensor as a game controller and motion-tracking sensor enhances home-based rehabilitation.

## 5. Conclusion

The smart elbow brace (SEB) model discussed above is a gadget that aids in elbow stiffness training outside the therapeutic environment. The advantage of this approach is that it offers the increased intensity of treatment and reduces in-patient while at the same time reducing rehabilitation costs. However, only patients who can safely move their elbow joint may be eligible for this type of therapy.

Mechanical design requirements such as standardization, mobilization, safety, wearable, portability, and simplicity of components met their requirements. Calculations of the device were established, and the device was designed. Furthermore, elbow stiffness serious games were developed. The MEMS IMU sensor as a motion-tracking sensor was considered due to its advantages over the other sensors, and such advantages were portability, fewer components, use of any place, being noninvasive, cost-effectiveness, accuracy, and availability. The sensor showed very high accuracy in detecting elbow joint motion.

However, this study has several limitations; for example, the effectiveness of the device was never quantified in clinical settings with elbow stiffness patients. Another limitation was weaker signals due to a Bluetooth module that makes a delayed action. During testing, users experienced that the speed of the elbow movement does not correlate precisely with the serious game movement. Moreover, the results after rehabilitation were saved in the user's personal computer, which can be lost.

Despite the proposed smart elbow brace proving its functional ability and be used at home as a complementary tool to support elbow stiffness rehabilitation during long-term home recovery, the following improvements to the SEB device's assessment and functionality will be considered in the future: (1) to quantify its effectiveness by involving elbow stiffness patients in rehabilitation, (2) to improve motion-tracking mechanisms by considering WiFi a means of communication to offer a wide range of control, (3) to improve motivation reward by considering 3D serious games development together with the development of a serious games library specific for different patients' interests and ages, and (4) reconsideration of the use of a web server. Whenever a patient trains, all data should be saved and accessed by the therapist directly from the server for further progress evaluation.

## Figures and Tables

**Figure 1:** 3D model of the designed SEB as a home-based rehabilitation device consists of 2-DoF.

**Figure 2:** Detailed design of a smart elbow brace.

**Figure 3:** A schematic diagram of the designed SEB operation.

**Figure 4:** Total weight required to be supported by the forearm splint.

**Figure 5:** Stopping mechanisms as angle adjusters.

**Figure 6:** Motion-tracking system electronic block design.

**Figure 7:** The IMU frames and Earth frames.

**Figure 8:** The ball-catching game (a) with the self-assessment avatar of a player (b). After the game setup, the avatar is turned on to see whether the sensor is in the right position and right elbow.

**Figure 9:** SEB was worn by a participant to test ROM and to use it for serious game rehabilitation.

**Figure 10:** Forearm stress analysis.

**Figure 11:** The angles and time attained by the participants when they were playing a serious game using SEB: (a) maximum and minimum angles attained from the flexion-extension rehabilitation and (b) maximum and minimum angles attained from the pronation-supination.

**Table 1:** Human anthropometric 95th percentile data (HAD).

Name	Male	Female
Length of the upper arm (m)	0.39	0.36
Hand length (upper arm + forearm) (m)	0.52	0.46
Mass in the lower arm (kg)	1.66	1.24
Upper arm mass (kg)	2.67	2.07
Position of lower arm and hand center of mass (%)	0.318	
Bicep's circumference, relaxed (cm)	35.1	29.3
Bicep's circumference, flexed (cm)	36.9	—
Forearm circumference, relaxed (cm)	32.7	24.1
Wrist circumference (cm)	19.3	16.2
Elbow width (cm)	8.2	7.4

**Table 2:** The relationship between designed SEB and normal human ROM.

Type of ROM	Normal human ROM in degrees (90% of normal daily activity)	Designed elbow brace ROM in degrees
Elbow flexion/extension	130/30	135/0
Forearm pronation/supination	50/50	50/50

## Data Availability

The data can be found by emailing the corresponding author.

## References

[1] Sojbjerg J. O. (1996). The stiff elbow: how I do it. *Acta Orthopaedica Scandinavica*.

[2] Murray O., Macdonald D., Nunn T., Mceachan J., Rymaszewski L. (January. 2012). Management of the post-traumatic stiff elbow. *Shoulder & Elbow*.

[3] Anastasios Papadonikolakis M. (2017). Post-traumatic stiffness and malunion after supracondylar humerus fracture in an adolescent patient. *Shoulder and Elbow Surgrey*.

[4] Jupiter J. B., O’Driscoll S. W., Cohen M. S. (2003). The assessment and management of the stiff elbow. *Instr Course Lect*.

[5] Van Meulen F. B., Klaassen B., Held J. (January, 2016). Objective evaluation of the quality of movement in daily life after stroke. *Frontiers in Bioengineering and Biotechnology*.

[6] Adolfsson L. (2018). Post-traumatic stiff elbow. *EFORT Open Reviews*.

[7] Officer P., Professor A., Professor A. (2009). Stiff elbow bhavuk garg MS, MRCS, aman dua MS, vijay sharma MS, P P kotwal MS. *FAMS, FIMSA*.

[8] Morrey B. F., Askew L. J., Chao E. Y., Chao E. Y. (1981). A biomechanical study of normal functional elbow motion. *The Journal of Bone and Joint Surgery*.

[9] Jones V. (April, 2016). Conservative management of the post-traumatic stiff elbow: a physiotherapist’s perspective. *Shoulder & Elbow*.

[10] Filh G. M., Galvão M. V. (July. 2010). POST-TRAUMATIC stiffness OF the elbow. *Revista Brasileira de Ortopedia (English Edition)*.

[11] Fusaro I., Orsini S., Sforza T., Rotini R., Benedetti M. (2014). The use of braces in the rehabilitation treatment of the post-traumatic elbow. *Joints*.

[12] Wang Q., Markopoulos P., Yu B., Chen W., Timmermans A. (March, 2017). Interactive wearable systems for upper body rehabilitation: a systematic review. *Journal of NeuroEngineering and Rehabilitation*.

[13] Wang S.-H., Zhang Y.-D. (June, 2020). DenseNet-201-Based deep neural network with composite learning factor and precomputation for multiple sclerosis classification. *ACM Transactions on Multimedia Computing, Communications, and Applications*.

[14] Yin, Xu H.-M. A wearable rehabilitation game controller using IMU sensor.

[15] Kadir K., Yusof Z. M., Rasin M. Z. M., Billah M. M., Salikin Q. Wireless IMU: a wearable smart sensor for disability rehabilitation training.

[16] Howard A., Brooks D., Brown E., Gebregiorgis A., Chen Y. P. Non-contact versus contact-based sensing methodologies for in-home upper arm robotic rehabilitation.

[17] Kyrylova A. (2015). *Development of a Wearable Mechatronic Elbow Brace for Postoperative Motion Rehabilitation*.

[18] Hsieh Y. W., Chang K. C., Hung J. W., Wu C. Y., Fu M. H., Chen C. C. (2018). Effects of home-based versus clinic-based rehabilitation combining mirror therapy and task-specific training for patients with stroke: a randomized crossover trial. *Archives of Physical Medicine and Rehabilitation*.

[19] Lee I. F.-K., Yau F. N., Yim S. S.-H., Lee D. T.-F. (2018). Evaluating the impact of a home-based rehabilitation service on older people and their caregivers: a matched-control quasi-experimental study. *Clinical Interventions in Aging*.

[20] Rahimi-Movaghar V., Rezaei M., Sharifi A., Vaccaro A. (2019). Home-based rehabilitation programs: promising field to maximize function of patients with traumatic spinal cord injury. *Asian Journal of Neurosurgery*.

[21] López-Liria R., Padilla-Góngora D., Catalan-Matamoros D., Rocamora-Pérez P., Pérez-de la Cruz S., Fernández-Sánchez M. (2015). Home-based versus hospital-based rehabilitation program after total knee replacement. *BioMed Research International*.

[22] Wang S.-H., Zhang Y.-D., Yang M., Liu B., Ramirez J., Gorriz J. M. (September. 2019). Unilateral sensorineural hearing loss identification based on double-density dual-tree complex wavelet transform and multinomial logistic regression. *Integrated Computer-Aided Engineering*.

[23] Laamarti F., Eid M., Saddik El (2014). An overview of serious games. *International Journal of Computer Games Technology*.

[24] Hoffman B., Nadelson L. (June. 2010). Motivational engagement and video gaming: a mixed methods study. *Educational Technology Research & Development*.

[25] Imam B., Miller W. C., Finlayson H. C., Eng J. J., Jarus T. (2018). A clinical survey about commercial games in lower limb prosthetic rehabilitation. *Prosthetics and Orthotics International*.

[26] Bonnechère B., Jansen B., Omelina L., Van Sint Jan S. (2016). The use of commercial video games in rehabilitation: a systematic review. *International Journal of Rehabilitation Research*.

[27] Voon K., Silberstein I., Eranki A., Phillips M., Wood F. M., Edgar D. W. (2016). Xbox Kinect based rehabilitation as a feasible adjunct for minor upper limb burns rehabilitation: a pilot RCT. *Burns*.

[28] McNulty P., Mouawad M., Doust C., Max M. (May 2011). Wii-based movement therapy to promote improved upper extremity function post-stroke: a pilot study. *Journal of Rehabilitation Medicine*.

[29] Yong Joo L., Soon Yin T., Xu D., Thia E., Pei Fen C., Kuah C. W., Kong K. H. (May 2010). “A feasibility study using interactive commercial off-the-shelf computer gaming in upper limb rehabilitation in patients after stroke. *Journal of Rehabilitation Medicine*.

[30] Zhang Y. D., Dong Z., Wang S. H. (December, 2020). Advances in multimodal data fusion in neuroimaging: overview, challenges, and novel orientation. *Information Fusion*.

[31] Lisini Baldi T., Farina F., Garulli A., Giannitrapani A., Prattichizzo D. (January. 2020). Upper body pose estimation using wearable inertial sensors and multiplicative kalman filter. *IEEE Sensors Journal*.

[32] Zhang Y.-D., Satapathy S. C., Guttery D. S., Górriz J. M., Wang S.-H. (2021). Improved breast cancer classification through combining graph convolutional network and convolutional neural network. *Information Processing & Management*.

[33] Huston R. L. (2009). *Principles of Biomechanics*.

[34] McConville J. (2018). Anthropometric relationships of body and body segments moments of inertia. *Anthropometry and Biomechanics*.

[35] Masjedi M., Duffell L. D. (2013). Dynamic analysis of the upper limb during activities of daily living: comparison of methodologies. *Proceedings of the Institution of Mechanical Engineers - Part H: Journal of Engineering in Medicine*.

[36] Bhat A., Janarthanan M. (2017). Human joint anatomy and physiology. *Sawhney, S., Aggarwal, A, Pediatric Rheumatology*.

[37] Kai-Nan An B. F. M., Zobitz M. E. (2017). Biomechanics of the elbow. *Clinicalgate.Orthopaedics*.

[38] Brinckmann P., Drerup B, Kretschmer T, Schulze-Frenking D, Wohlatz A, Wetz H. H (March. 2007). Locating the Axis of rotation when fitting an elbow orthosis. *Prosthetics and Orthotics International*.

[39] Deland J. T., Garg A., Walker P. S. (1997). Biomechanical basis for elbow hinge-distractor design. *Clinical Orthopaedics and Related Research*.

[40] Ang W. S., Chen I. M., Yuan Q. Ambulatory measurement of elbow kinematics using inertial measurement units.

[41] Yuan Q., Chen I. M., Lee S. P. SLAC: 3D localization of human based on kinetic human movement capture.

[42] I-Ming Chen Q., Chen I.-M. Simultaneous localization and capture with velocity information.

